# miR-134-5p promotes inflammation and apoptosis of trophoblast cells via regulating FOXP2 transcription in gestational diabetes mellitus

This article has been retracted.

**DOI:** 10.1080/21655979.2021.2001219

**Published:** 2021-12-30

**Authors:** Weiqi Ke, Yixiang Chen, Lijing Zheng, Yuting Zhang, Yudan Wu, Li Li

**Affiliations:** a Department of Anesthesiology, The First Affiliated Hospital of Shantou University Medical College, Shantou, Guangdong Province, China; b Department of Gynecology and Obstetrics, The First Affiliated Hospital of Shantou University Medical College, Shantou, Guangdong Province, China

**Keywords:** miR-134-5p, FOXP2, gestational diabetes mellitus, apoptosis, inflammation, high glucose

## Abstract

Gestational diabetes mellitus (GDM) is a prevalent and risky pregnant complication which warrants targeted therapy for restriction the inflammation and apoptosis of trophoblast cells. This study sought to analyze the aberrant expression and regulatory mechanism of microRNA (miR)-134-5p in GDM. The miR-134-5p expression in the serum of GDM patients and normal participants was detected via qRT-PCR, followed by receiver operating characteristic (ROC) curve analysis. *In vitro* GDM cell model was established in the HTR-8/SVneo cells using 25 mmol/L glucose, followed by transfection with miR-134-5p inhibitor and si-Forkhead box p2(FOXP2). The miR-134-5p and FOXP2 expressions, TNF-α, IL-1β, and IL-10 levels, cell proliferation, migration, and apoptosis were determined by a combination of qRT-PCR, western blot, ELISA, and cell counting Kit-8, Transwell assay, and flow cytometry. The binding relationship between miR-134-5p and FOXP2 was predicted and verified. Our results revealed that miR-134-5p was increased in the serum of GDM patients and could serve as a critical diagnostic marker for GDM. Moreover, miR-134-5p was upregulated in the high glucose (HG)-induced HTR-8/SVneo cells. The miR-134-5p inhibition suppressed the inflammation and apoptosis of HG-induced HTR-8/SVneo cells. miR-134-5p inhibited FOXP2 expression. FOXP2 expression was decreased in GDM. FOXP2 inhibition attenuated the function of miR-134-5p in HG-induced HTR-8/SVneo cells. Overall, miR-134-5p inhibited the FOXP2 expression to facilitate the inflammation and apoptosis of trophoblast cells, thereby exacerbating GDM.

## Introduction

Gestational diabetes mellitus (GDM) is regarded as the most prevalent pregnancy complication, clinically manifested due to abnormal glucose intolerance and fasting glucose (≥92 mg/dL) that precipitates to chronic hyperglycemia and threatens safe pregnancy [1,2]. GDM is a dangerous condition for both mothers and infants as it amplifies the associated risks of antenatal depression, preterm birth, preeclampsia, fetal overgrowth, neonatal hypoglycemia, and several others [1]. The development of trophoblasts (the outer layer of the placenta) is essential for a successful pregnancy and is involved in the pathophysiology of multiple gestational diseases [3]. Previously, hyperglycaemic condition in GDM can evidently evoke a pro-inflammatory response in trophoblasts, thus exacerbation the degree of apoptosis of trophoblast cells [4]. The currently available treatments for the management of hyperglycemia fundamentally repair the inflammatory insult and trophoblast dysfunction induced by GDM [5,6]. However, drug therapeutics for the management of hyperglycemia present with varying degrees of maternal and infant complications, depending on factors such as age, physical condition, pregnancy stage, and complications [7] Therefore, the development of targeted methods is necessitated for the management of inflammation and apoptosis in trophoblasts for GDM treatment.

MicroRNAs (miRNAs) are a class of small noncoding RNAs (21–25 nucleotides) with vital functionality in the epigenetic regulation of GDM [8]. Previously, miR-134 has been identified as a critical component in endothelial cell dysfunction in diabetes and inflammation in conditions such as atherosclerosis and Hepatitis C Virus [9–11]. Essentially, miR-134-5p has been identified as a potential diagnostic marker of GDM [12]. Extensive research has highlighted the role of miR-134-5p in cellular metabolism, particularly the proliferation, migration, and apoptosis of cancer cells [13,14]. Notably, an existing study demonstrated the ability of miR-134-5p to regulate trophoblast cell behaviors in preeclampsia, such as apoptosis, migration, and invasion [15]. Nevertheless, the molecular mechanism of miR-134-5p in GDM remains elusive.

Moreover, a prior study identified that miR-134-5p can target Forkhead box protein 2 (FOXP2) in early vascular dementia [16]. FOXP2 is a highly conserved transcription factor that functions as a definitive regulator of embryonal development with human speech and language [17]. An existing research unveiled that FOXP2 was downregulated in hyperglycemia and it enhances the cell viability, proliferation, and migration of high glucose (HG)-induced human microvascular endothelial cells, thereby attenuating and relieving diabetes symptoms [18,19]. Additionally, FOXP2 elicits suppressive functionality in the apoptosis and inflammation of several types of cells, such as neurons, cardiomyocytes, and lymphoma [20–22]. Moreover, the role of FOXP2 in trophoblast cell function and the interaction between miR-134-5p and FOXP2 in GDM remain unidentified.

In light of the aforementioned literature, we hypothesized that miR-134-5p could regulate the inflammation and apoptosis in trophoblast cells via targeting FOXP2. On the basis of this hypothesis and detection of clinical samples, we established an *in vitro* cell model to evaluate the therapeutic role of miR-134-5p/FOXP2 in trophoblast cell dysfunction, hoping to provide a targeted protocol for GDM treatment.

## Materials and methods

### Ethics statement

The current study was conducted with approval of the Ethics Committee of The First Affiliated Hospital of Shantou University Medical College. All participants provided informed signed consent prior to participation.

### Experimental subjects

A total of 140 individually were enrolled in this study, namely 70 GDM patients and 70 healthy pregnant women as controls from a period from March 2018 to December 2019 in The First Affiliated Hospital of Shantou University Medical College. All participants underwent an oral glucose tolerance test during the 24–28th week of gestation. Fasting serum samples were collected from participants and preserved at −80°C.

### *Standards of gestational diabetes mellitus diagnosis* [23]

GDM patients were diagnosed using the standards provided by the American Diabetes Association. At 24–28 weeks of gestation, the pregnant women took glucose solution (75 g glucose dissolved in 300 mL water) at least 8 h after fasting, followed by measurement of glucose concentration in venous blood using the glucose oxidase method in fasting state, and glucose concentration at 1 and 2 h after administration of glucose solution. GDM was verified with multiple abnormalities: fasting glucose ≥92 mg/dl (5.1 mmol/L); 1-h glucose ≥180 mg/dl (10.0 mmol/L); 2-h glucose ≥153 mg/dl (8.5 mmol/L). The exclusion criteria for the patients was as follows: multiple pregnancies; diabetes prior to pregnancy; gestational hypertension; eclampsia; malignancy, acute or chronic infectious diseases; hypertension; rheumatic diseases; liver cirrhosis; congestive heart failure; gout and other endocrine metabolic diseases.

### *Cell culture and transfection* [24]

Trophoblast cell lines HRT-8/SVneo (ATCC, Manassas, VA, USA) were pre-cultured using Roswell Park Memorial Institute 1640 medium (Invitrogen, Carlsbad, CA, USA) supplemented with 10% fetal bovine serum (Thermo Fisher Scientific, Waltham, MA, USA) at 37°C with 5% CO_2_. Next, the HRT-8/SVneo cells were classified into the HG group and the control group [normal glucose (NG) group]. HRT-8/SVneo cells in the HG group were incubated in HG medium (containing 25 mM glucose) and the cells in the control group were cultured in medium containing 5 mM of glucose [25]. After completion of cell passage, they were detached with trypsin (15090046, Thermo Fisher Scientific). Subsequently, the HRT-8/SVneo cells in the HG medium were transfected with the miR-134-5p inhibitor, inhibitor NC, si-FOXP2, or si-NC (Shanghai GenePharma Co., Ltd, Shanghai, China) using Lipofectamine 2000. After 48 h, the transfected cells were isolated for subsequent experimentation. All experiments were conducted 3 times independently.

### *Reverse transcription quantitative polymerase chain reaction (qRT-PCR)* [12]

The total RNA content was extracted from the serum samples and cells and reverse-transcribed into complementary DNA (cDNA) using the TRlzol reagent (Invitrogen) and the reverse transcription kit (RR047A, Takara, Tokyo, Japan). Next, for the detection of miRNA, the RNA content was reverse transcribed into cDNA using the miRcute miRNA First-Strand cDNA Synthesis kit (TianGen, Beijing, China). Subsequently, qRT-PCR assay was conducted using SYBR Premix EX Taq^TM^ II (Tli RAaseH Plus) (Takara, Dalian, China) in a fluorescent quantitative PCR device (ABI 7500, ABI, Foster City, CA, USA). PCR was amplified in compliance with the following procedure: pre-treatment at 95°C for 30 s, followed by 40 cycles of samples at 95°C for 5 s, at 60°C for 34 s, and extension at 95°C for 15 s. Each sample was provided with three duplicated wells. The PCR primers were synthesized by Sangon Biotech (Shanghai, China) Co., Ltd (shown in Table 1). Ct value of each well was documented and relative gene expression was estimated based on the 2^−ΔΔCt^ method with GAPDH or U6 as the internal reference.

**Table 1.** qPCR primers

Gene	Forward Primer (5ʹ-3ʹ)	Reverse Primer (5ʹ-3ʹ)
miR-134-5p	GCCGAGGGGGAGACCAGUUG	CTCAACTGGTGTCGTGGA
FOXP2	GAAGACAATGGCATTAAACATGGAGG	GAATAAAGCTCATGAGATTTACCTGTC
TNF-α	ATGTGGCAAGAGATGGGGAA	CTCACACCCCACATCTGTCT
IL-1β	CACGATGCACCTGTACGATCA	GTTGCTCCATATCCTGTCCCT
IL-10	CTACTAAGGCTTCTTTGGGAG	CTACTAAGGCTTCTTTGGGAG
BCL-2	GGAGAGCGTCAACAGGGAGA	CAGCCAGGAGAAATCAAACAGAG
Bax	TTCTGACGGCAACTTCAACT	CAGCCCATGATGGTTCTGAT
GAPDH	CAGTCACTACTCAGCTGCCA	TGGTGAAGACGCCAGTGGA
U6	CTCGCTTCGGCAGCACA	AACGCTTCACGAATTTGCGT

### *Western blotting* [26]

The total protein content was extracted from the HTR8/SVneo cells at 4°C using the RIPA buffer (Beyotime Institute of Biotechnology, Shanghai, China). The protein concentration was quantified using the bicinchoninic acid assay kit (Beyotime Institute of Biotechnology). Next, the proteins (30 g/lane) were isolated using 10% sodium dodecyl sulfate polyacrylamide gel electrophoresis and transferred onto polyvinylidene fluoride membranes. Subsequently, a membrane blockade was conducted using 5% skim milk containing Tween 20 (TBST) for 1.5 h. Next, the membranes were subject to incubation with anti-FOXP2 (at a dilution ratio of 1:1000, ab172320, Abcam) and GAPDH (at a dilution ratio of 1:1000, ab8245, Abcam). After a rinse with TBST, the membranes were incubated with the corresponding horseradish peroxidase-labeled secondary antibody (at a dilution ratio of 1:5000, ab6759, Abcam) for 2 h. The protein bands were visualized using the enhanced chemiluminescence kit (Applygen Technologies, Inc., Beijing, China). The protein expression pattern was determined using the ImageJ software, with GAPDH as internal reference.

### *Cell counting kit-8 (CCK-8)* [27]

After cell transfection, the cells were seeded into 96-well plates, with subsequent addition of the CCK-8 solution at 24, 36, 48, and 60 h. Next, the absorbance value at the excitation wavelength of 450 nm was determined using a microplate reader (Bio-Rad 680, Hercules, CA, USA) to assess the cell proliferative rate.

### *Transwell assay* [25]

At 48 h after cell transfection, the cells were cultured with serum-free RPMI 1640 medium to isolate the cell suspension. The 200 μL cell suspension and 800 μL RPMI 1640 medium [containing 10% phosphate buffer saline (PBS)] were respectively added into the apical chamber and basolateral chamber for a 24 h-incubation regimen at 37°C with 5% CO_2_. Next, the migrated cells were fixed in 4% paraformaldehyde and stained using 1% crystal violet (Sigma-Aldrich, MO, USA). The cells were counted under a microscope from 5 random visual fields.

### *Enzyme-linked immunosorbent assay (ELISA)* [28]

At 48 h after cell transfection, the supernatants of all groups were isolated. The levels of tumor necrosis factor (TNF)-α, interleukin (IL)-1β, and IL-10 were determined using the ELISA kits (R&D Systems, Minneapolis, MN, USA).

### *Flow cytometry* [13]

Meanwhile, the cells were stained with fluorescein isothiocyanate (FITC) and propidium iodide (PI) in strict accordance with the provided instructions of the Annexin V-FITC kits (BioVision, Bay Area, SF, USA). Next, 1 × 10^5^ cells were rinsed with PBS twice and re-suspended using 100 μL of binding buffer, followed by the addition of 2 μL Annexin V-FITC solution and 15 min-incubation on ice in conditions devoid of light. Next, the cells were supplemented with 400 μL PBS and 1 μL PI. The apoptotic cells were detected using the flow cytometer (Invitrogen, Thermo Fisher Scientific)

### *Dual-luciferase reporter assay* [29]

The potential binding sites of miR-134-5p and FOXP2 were predicted using the TargetScan website (http://www.targetscan.org/). Next, FOXP2 3ʹ-UTR wildtype (WT) and mutant type (MUT) sequences were inserted into the luciferase vector pmiR-Report (Ambion, Grand Island, NY, USA) to successfully construct FOXP2-WT and FOXP2-MUT plasmids. Next, the preceding plasmids and miR-134-5p mimic/mimic NC were co-transfected into the HEK-293 T cells (ATCC). After 48 h, the cells were harvested, followed by detection of luciferase activity.

### Statistical analysis

SPSS21.0 software (IBM Corp, Armonk, NY, USA) and GraphPad Prism 8.0 software (GraphPad Software Inc., San Diego, CA, USA) were adopted for data analysis and graphing. Enumeration data were represented as case numbers and percentages. The pairwise comparisons were analyzed using the chi-square test. The measurement data were represented as mean ± standard deviation (SD) with normal distribution and homogeneity of variance. The pairwise comparisons and comparisons among multiple groups were analyzed respectively using the *t* test and one-way or two-way analysis of variance (ANOVA), followed by Tukey’s multiple comparison test. A *P* value was obtained from the two-tailed tests. In all statistical references, a value of *P* < 0.05 was indicative of statistical significance.

## Results

The current study sought to explore the abnormal expression pattern of miR-134-5p in GDM and the role of miR-134-5p in the inflammation and apoptosis of trophoblast cells. Initially, we analyzed the clinical baseline data of GDM patients and evaluated the correlation between miR-134-5p and fasting glucose using the receiver operator characteristic (ROC) curve to verify the diagnostic value of miR-134-5p in GDM. Subsequently, we established *in vitro* GDM model via the HG inducing HTR8/SVneo cells, and transfection of miR-134-5p inhibitor was conducted to evaluate the role of miR-134-5p in the proliferation, migration, inflammation, and apoptosis of HTR8/SVneo cells. Next, we speculated the role of FOXP2 as a downstream target of miR-134-5p and downregulated FOXP2 in HTR8/SVneo cells for the rescue experiment.

### Clinical characteristics of the study population

Among the enrolled study subjects, parameters such as maternal age and gestational age at delivery of GDM patients and normal pregnant women had no statistical difference (*P* > 0.05). However, parameters such as body mass index (BMI), fasting glucose, 1 h-glucose, 2 h-glucose, infant weight, fasting insulin, systolic pressure (SBP), diastolic pressure (DBP), and glycosylated hemoglobin (HbA1c) of GDM patients were markedly higher relative to the normal pregnant women (Table 2) (*P* < 0.05).

**Table 2.** Baseline characteristics of participants

Index	Normal	GDM	*P* Value
Maternal age (Years)	30.04 ± 2.25	30.33 ± 2.25	0.454
Gestational age at delivery (weeks)	38.76 ± 1.06	39.12 ± 1.15	0.056
Pre-pregnancy BMI (kg/m^2^)	22.51 ± 0.71	23.12 ± 2.30	**0.036**
Fasting glucose (mmol/L)	4.17 ± 0.19	6.31 ± 0.27	**0.001**
1h glucose (mmol/L)	6.02 ± 0.63	10.59 ± 0.66	**0.001**
2h glucose (mmol/L)	5.15 ± 0.51	9.12 ± 0.54	**0.001**
Infant weight (g)	3178.55 ± 126.27	3265.51 ± 154.25	**0.001**
Fasting insulin (mlU/L)	8.03 ± 0.90	8.54 ± 1.07	**0.001**
SBP (mmHG)	115.74 ± 11.51	119.73 ± 10.59	**0.034**
DBP (mmHG)	76.65 ± 9.84	80.67 ± 9.46	**0.015**
HbA1c (%)	5.09 ± 0.24	5.42 ± 0.20	**0.001**

BMI: body mass index; SBP: Systolic pressure; DBP: Diastolic pressure; HbA1c: Glycosylated hemoglobin

### miR-134-5p served as a potential diagnostic marker for gestational diabetes mellitus

Previous research has demonstrated that an early GDM diagnosis can influence the outcome of gestation, and miR-134 is associated with high GDM morbidity [12]. Hence, the miR-134-5p expression pattern in the serum of GDM patients was detected via qRT-PCR and the results showed that miR-134-5p was markedly upregulated in the serum of GDM patients compared to the normal pregnant women (*P* < 0.001, Figure 1(a)), thus indicating the participation of miR-134-5p in the GDM occurrence. To verify whether miR-134-5p could serve as a diagnostic marker for GDM, we plotted the ROC curve. The result showed that area under the ROC curve (AUC) was 0.7955, the sensitivity was 77% while the specificity was 70% (Figure 1(b)). Next, the Spearman correlation analysis showed that relative expression pattern of miR-134-5p was positively correlated with fasting glucose (Figure 1(c)). Altogether, our findings identified an explicit correlation between miR-134-5p and GDM occurrence and hence could serve as a potential diagnostic marker for GDM.

**Figure 1.** **miR-134-5p expression in the serum and analysis of receiver operator characteristic (ROC) curve**. (a) miR-134-5p expression pattern in the serum was detected via qRT-PCR, Normal (N = 70), GDM (N = 70); (b) ROC curve analysis, the area under the ROC curve (AUC) = 0.7955, *P* < 0.001; (c) Spearman correlation analysis of serum miR-134-5p in GDM patient and fasting glucose. Data in figure a was analyzed using *the t* test, followed by Tukey’s multiple comparison test. *** *P* < 0.001; GDM: gestational diabetes mellitus.

### High glucose (HG) improved miR-134-5p expression and downregulation of miR-134-5p promoted HG-induced proliferation and migration of trophoblast cells

To further explore the role of miR-134-5p in GDM, the HTR8/SVneo cells were cultured with HG to simulate GDM *in vitro*. Our results showed that after HG induction, the miR-134-5p expression pattern was increased (*P* < 0.05, Figure 2(a)), the cell viability was reduced (*P* < 0.05, Figure 2(b)), and the cell migration was diminished (*P* < 0.05, Figure 2(c)). Next, we downregulated the miR-134-5p expression pattern in HTR8/SVneo cells (*P* < 0.05, Figure 2(a)). Our results demonstrated that miR-134-5p downregulation facilitated the proliferation and migration of HG-induced HTR8/SVneo cells (*P* < 0.05, Figure 2(b-c))

**Figure 2.** **miR-134-5p was poorly expressed in HG-induced trophoblast cells and promoted proliferation and migration**. HTR8/SVneo cells were treated with 25 mM glucose with 5 mM glucose-treated cells as the control. (a) miR-134-5p expression pattern in different groups was detected via qRT-PCR; (b) Proliferation potential in different groups was detected via CCK-8; (c) Migration potential in different groups was detected via Transwell assay. Cell experiment was conducted 3 times and data were represented as mean ± SD. Data in figures a and c were analyzed using one-way ANOVA and data in figure b were analyzed using two-way ANOVA. After analysis, data were checked by Tukey’s multiple comparison test. *** *P* < 0.001; NG: normal glucose; HG: high glucose.

### Downregulation of miR-134-5p suppressed inflammation and apoptosis of high glucose-induced trophoblast cells

An existing study determined the critical functionality of cell inflammation and apoptosis in the initiation and progression of GDM [30]. To evaluate the effects of miR-134-5p on the inflammation and apoptosis of trophoblast cells in GDM patients, we detected the cytokine levels in different groups of HTR8/SVneo cells. Our results showed that HG induction elevated the TNF-α and IL-1β levels while it simultaneously reduced the IL-10 level, and miR-134-5p inhibition reduced the TNF-α and IL-1β levels alongside elevating the IL-10 level (*P* < 0.05, Figure 3(a,b)). Moreover, flow cytometry revealed that HG induction facilitated the apoptosis of HTR8/SVneo cells, whereas miR-134-5p inhibition suppressed the apoptosis of HTR8/SVneo cells (*P* < 0.05, Figure 3(c)), and the results of qRT-PCR showed that miR-134-5p inhibition suppressed the Bax expression pattern and markedly increased the Bcl-2 expression pattern (*P* < 0.05, Figure 3(d)). The preceding results elucidated the functionality of miR-134-5p in the inflammation and apoptosis of HG-induced HTR8/SVneo cells.

**Figure 3.** **miR-134-5p inhibition suppressed inflammation and apoptosis of trophocytes**. HTR8/SVneo cells were treated with 25 mM glucose, followed by transfection of miR-134-5p inhibitor with inhibitor NC as the control. TNF-α, IL-1β, and IL-10 levels were detected via qRT-PCR (a) and ELISA (b); (c) Cell apoptosis was detected via flow cytometry; (d) Bax and Bcl-2 expression patterns were detected via qRT-PCR. Cell experiment was conducted 3 times and data were represented as mean ± SD. Data in figures c and d were analyzed using one-way ANOVA and data in figures a and b were analyzed using two-way ANOVA. After analysis, data were checked by Tukey’s multiple comparison test. * *P* < 0.05, ** *P* < 0.01; *** *P* < 0.001; NG: normal glucose; HG: high glucose.

### miR-134-5p inhibited FOXP2 expression

Previously, FOXP2 has elicited involvement in the pathogenesis of diabetes [19] and can also inhibit cardiomyocyte apoptosis [21]. Prediction by the TargetScan website identified FOXP2 as a potential target of miR-134-5p, which was further validated by dual-luciferase reporter assay (*P* < 0.05, Figure 4(a)). Next, the FOXP2 expression patterns in the serum of normal pregnant women and GDM patients were detected. Our results elicited a poor expression pattern of FOXP2 in the serum of GDM patients (*P* < 0.05, Figure 4(b)) with a negative correlation with miR-134-5p (*P* < 0.05, Figure 4(c)). Moreover, the FOXP2 expression pattern was reduced in the HG-induced HTR8/SVneo cells and elevated after miR-134-5p downregulation (*P* < 0.05, Figure 4(d-e)). In conclusion, our results revealed that miR-134-5p inhibited the FOXP2 expression in GDM.

**Figure 4.** **miR-134-5p inhibited FOXP2 expression. (**a) Binding relationship between FOXP2 and miR-134-5p was verified via dual-luciferase reporter assay; (b) FOXP2 expression pattern in the serum was detected via qRT-PCR; (c) Correlation between FOXP2 and miR-134-5p was evaluated via Spearman correlation analysis; (d-e) FOXP2 expression pattern in trophoblast cells of different groups was detected via qRT-PCR and western blot analysis. Cell experiment was conducted 3 times and data was represented as mean ± SD. Data in figure B were analyzed using *t* test, data in figure d were analyzed using one-way ANOVA and data in figure a were analyzed using two-way ANOVA. After analysis, data were checked by Tukey’s multiple comparison test. * *P* < 0.05, ** *P* < 0.01; *** *P* < 0.001; GDM: gestational diabetes mellitus; NG: normal glucose; HG: high glucose.

### Silencing of FOXP2 reversed the effects of miR-134-5p downregulation on inhibiting inflammation and apoptosis in high glucose-induced trophoblast cells

To further determine the role of FOXP2 in the inflammation and apoptosis in GDM, the miR-134-5p inhibitor-treated HTR8/SVneo cells were transfected with si-FOXP2 (*P* < 0.05, Figure 5(a-b)). Our findings revealed that FOXP2 downregulation attenuated the effects of miR-134-5p inhibitor on restricting the release of TNF-α and IL-1β and increasing the release of IL-10 (*P* < 0.05, Figure 5(c-d)), and FOXP2 downregulation annulled the effects of miR-134-5p inhibitor on suppressing the apoptosis of HG-induced HTR8/SVneo cells (*P* < 0.05, Figure 5(e-f)). Overall, the results illustrated that miR-134-5p inhibited FOXP2 transcription to promote the inflammation and apoptosis in trophoblast cells.

**Figure 5.** **Silencing of FOXP2 reversed the inhibitory effects of miR-134-5p downregulation on inflammation and apoptosis in trophoblast cells**. HTR8/SVneo cells with downregulation of miR-134-5p were transfected with si-FOXP2 with si-NC as the control. (a-b) FOXP2 expression pattern in the trophoblast cells was detected via qRT-PCR and western blot analysis; TNF-α, IL-1β, and IL-10 levels were detected via qRT-PCR (c) and ELISA (d); (e) Cell apoptosis was detected via flow cytometry; F: Bax and Bcl-2 expression patterns were detected via qRT-PCR. Cell experiment was conducted 3 times and data were represented as mean ± SD. Data in figures A, B, D, E and F were analyzed using one-way ANOVA and data in figures c and d were analyzed using two-way ANOVA. After analysis, data were checked by Tukey’s multiple comparison test. * *P* < 0.05, ** *P* < 0.01; *** *P* < 0.001; HG: high glucose.

## Discussion

GDM is a dangerous condition during pregnancy that progresses to inflammation and apoptosis in the trophoblast [4]. Recently, the functionality of miR-134-5p has been identified as a potential diagnostic marker of GDM with notable function in the regulation of trophoblast cell metabolism [12,15]. Accumulating evidence has highlighted that FOXP2is targeted by miR-134-5p and can explicitly manipulate cellular in diabetes [16,19]. In the current study, we illustrated that miR-134-5p inhibits FOXP2 transcription to promote the inflammation and apoptosis of HG-treated HTR8/SVneo cells (Figure 6).

**Figure 6.** **Mechanism of miR-134-5p in inflammation and apoptosis of trophoblast cells**. miR-134-5p inhibits the FOXP2 expression pattern to promote the inflammation and apoptosis of HG-treated HTR8/SVneo cells.

Initially, we analyzed the clinical characteristics of the study population to validate that certain representative characteristics (BMI, fasting glucose, 1 h-glucose, 2 h-glucose, infant weight, fasting insulin, SBP, DBP, and HbA1c)) of GDM patients were higher relative to the normal pregnant women. Next, our findings revealed an elevated miR-134-5p expression in the serum of GDM patients, which is consistent with existing research eliciting that miR-134-5p is elevated in GDM women [12]. Next, the ROS analysis revealed that the area under the ROC curve of miR-134-5p was 0.7955, with 77% sensitivity and 70% specificity. Spearman correlation analysis identified a positive correlation between the miR-134-5p expression and fasting glucose. The preceding results elucidated that miR-134-5p could serve as a potential diagnostic marker of GDM.

To further explore the fundamental role of miR-134-5p in GDM, the HTR8/SVneo cells were treated with 25 nM glucose to simulate GDM *in vitro*, followed by transfection with the miR-134-5p inhibitor. Proliferative and migration properties are fundamental for continuous growth of trophoblast cells, thus radically affecting the development of GDM [31]. HG induction increased the miR-134-5p expression and reduced the cell viability, proliferation, and migration, while miR-134-5p inhibition facilitated cell proliferation and migration. Consistently, the miR-134 inhibitor could evidently weaken the invasiveness of trophoblast cells and loss of miR-134-5p could exacerbate the proliferation and migration of trophoblast cells in preeclampsia [15,32]. Collectively, our findings elicited that miR-134-5p downregulation enhances the cell proliferation and migration of trophoblast cells.

Moreover, extensive cell inflammation and apoptosis in trophoblasts are vital pathological findings of GDM [4]. Notably, TNF-α and IL-1β are pro-inflammatory cytokines and IL-10 is an anti-inflammatory cytokine in diabetes [33]. Furthermore, Bcl-2 has an inhibitory effect on apoptosis while Bax can excavate it in trophoblasts [34]. Our results illustrated that HG could elevate the release of TNF-α, IL-1β, and Bax and inhibit the release of IL-10 and Bcl-2, where miR-134-5p inhibition could annul molecular alternations, indicating that miR-134-5p had induced inflammation and apoptosis. Previously, an existing study demonstrated the capacity of miR-134-5p to induce the apoptosis of trophoblast cells in preeclampsia via down-regulation of Yes-associated protein 1 [15]. Moreover, miR-134 has been identified as an effective target that facilitates proinflammatory cytokine production in atherosclerosis [10]. Although a prior study demonstrated that miR-362-5p can modulate the proliferation and apoptosis of HTR8/SVneo cells [35], the role of certain miRNAs in trophoblast cells secreted-pro-inflammatory cytokine production remains elusive. Essentially, the pro-inflammatory property of miR-134-5p on trophoblast cells has not been identified. Altogether, our results demonstrated that miR-134-5p promotes the apoptosis and inflammation of trophoblast cells.

Subsequently, we analyzed the downstream mechanism of miR-134-5p. Through data prediction, FOXP2 was identified. Previous research determined the targeting relationship between miR-134-5p and FOXP2 in vascular dementia and reduction of FOXP2 in hyperglycemia [16,18]. In the current study, FOXP2 was verified as a definitive target of miR-134-5p via dual-luciferase reporter assay. Next, the results of qRT-PCR elicited a poor expression of FOXP2 in GSM patients with a negative correlation with miR-134-5p. Moreover, our findings determined a reduced FOXP2 transcriptional level in HG-induced HTR8/SVneo cells and with further modulation after miR-134-5p downregulation. To further evaluate the role of FOXP2 in GDM, si-FOXP2 was transfected into the HG-induced HTR8/SVneo cells with the downregulation of miR-134-5p. Moreover, FOXP2 inhibition could efficacious annul the suppressive role of miR-134-5p inhibitor in the inflammation and apoptosis of trophoblast cells. An existing study revealed that FOXP2 could radically improve the viability of human microvascular endothelial cells [19]. Consistently, FOXP2 overexpression inhibits the apoptosis in cardiomyocytes and lymphoma and attenuates the inflammation of neurons [20–22]. In light of existing literature, the effect of FOXP2 in trophoblast cells has not been research extensively. Overall, our study identified that the miR-134-5p increases FOXP2 transcription to function as a stimulant in the inflammation and apoptosis of trophoblast cells.

## Conclusion

To conclude, our results revealed that miR-134-5p is a vital component in mediating the inflammation and apoptosis of trophoblast cells via regulation of FOXP2 transcription. Therefore, this study is the first of its kind to demonstrate the interaction between miR-134-5p and FOXP2 in trophoblast cell dysfunction and speculated at the development of targeted protocol for GDM treatment. Although we verified the role of miR-134-5p in HG-induced trophoblast cells via targeting FOXP2, the current study was unable to investigate the effects of miR-134-5p on animals and regulation of other target genes. Additionally, the role of miR-134-5p/FOXP2 in other factors underlying GDM, such as glucose metabolism and insulin resistance warrants investigation. In the future, comprehensive animal experiments are warranted with upstream mechanisms and other targets of miR-134-5p in GDM, and the role of miR-134-5p/FOXP2 in glucose metabolism and insulin resistance also warrants investigation for a valuable insight for GDM treatment.
